The article "Outbound Data Legality Analysis in CPTPP Countries under the Environment of Cross-Border Data Flow Governance" was retracted in 2023. Reasons: unreliable results or conclusions; concerns about the data; concerns about the results or conclusions; concerns about the peer review.

# Outbound Data Legality Analysis in CPTPP Countries under the Environment of Cross-Border Data Flow Governance

**DOI:** 10.1155/2022/6105804

**Published:** 2022-09-28

**Authors:** Jing Li

**Affiliations:** School of Law, Xi'an Jiaotong University, Xi'an, Shaanxi 710000, China

## Abstract

The governance of cross-border data flows around the digital economy, data security, and data sovereignty has become a crucial global governance issue. This paper evaluates the legitimacy of data exit rules of CPTPP countries based on machine learning algorithm models under the perspective of cross-border data flow governance. In this study, four machine learning algorithms, namely, logistic regression, decision tree, random forest, and GBDT, are used to build an outbound data assessment and evaluation model. The confusion matrix is used to classify the outbound data legitimacy dichotomously. The recall, precision, and F1 scores are evaluated to compare the empirical results of each model. Based on this, a logistic regression-based outbound data risk scoring model is introduced to quantify the outbound data risk at a deeper level and to classify the outbound data risk level for the reference of regulators to make more scientific and reasonable decisions. The experimental results show that the machine learning models can meet the needs and applications of practical work and make accurate predictions of outbound data risks.

## 1. Introduction

The digital era with “data” as the core feature has arrived, and the new generation of information technology represented by digital technology has become the focus of the fourth industrial revolution. The interconnection of the Internet has led to the large-scale cross-border flow of data, which has penetrated various fields of political, economic, and social life [1]. In the economic aspect, the cross-border flow of data has replaced the flow of goods and capital as the primary trend of economic globalization. While cross-border data flow brings excellent economic value and social convenience, it also dramatically impacts data security and sovereignty [2]. With the rapid growth of cross-border data flow, data leakage incidents are frequent, and the data security of the state, citizens, and society is facing unprecedented threats. In addition, the high mobility of cross-border data raises new questions about the traditional concept of “sovereignty,” including how to determine the sovereignty of cross-border data and whether cross-border data flow poses a challenge to national security and social stability, which makes countries pay great attention to the cross-border data flow .

The governance of cross-border data flows around the digital economy, data security, and data sovereignty has become an essential issue of global governance [3]. However, countries have introduced relevant data governance policies as the international community has not yet reached uniform rules on cross-border data governance. However, differences in governance concepts and other aspects have led to a trend of increased conflict and contention in this area. How to share the dividends of cross-border data flow and promote the development of the digital economy while effectively maintaining data security and weakening the disputes over data sovereignty has become a pressing problem in the field of cross-border data flow governance.

The article "Outbound Data Legality Analysis in CPTPP Countries under the Environment of Cross-Border Data Flow Governance" was retracted in 2023. Reasons: unreliable results or conclusions; concerns about the data; concerns about the results or conclusions; concerns about the peer review.

This paper analyzes the legitimacy of CPTPP country exit rules from the perspective of cross-border data flow governance. It uses four machine learning algorithms, namely, logistic regression, decision tree, random forest, and GBDT, to determine the legitimacy of cross-border data.

## 2. Literature Review

### 2.1. Theory of Cross-Border Data Flow Governance

#### 2.1.1. Cross-Border Data

The information civilization that began in the last century has generated epoch-making changes such as computers and the Internet and has inspired new vitality, ushering in the creation and development of new technology clusters including cloud computing, mobile Internet, Internet of Things, artificial intelligence, and big data. Among these new technologies, data is the primary carrier of network information content and the basic material for production activities, and the essence of the Internet is the flow of data [4].

The era of “data” as a critical production factor driving economic and social innovation and development has arrived [5]. The flow of data across borders is increasingly replacing the flow of goods and capital as the primary trend of economic globalization. “Data” is essential for the development of national competitiveness.

“Data” should be defined as “information carriers designed to record the subjective reflection of the subject of knowledge on the object of knowledge”; mainly includes personal data, business data, technical data, and organizational data; and is essential, reproducible, and mobile [6].

Cross-border data refers to the flow of data across sovereign state borders through information technology, which refers to the flow of data across national borders or geographical boundaries through various technologies and methods. Cross-border data includes personal and nonpersonal data, such as confidential data related to national security, data held by governments, institutions, or enterprises, intellectual property data, and digital products [7].

It can be seen that data are usually generated within a country and have the potential to flow across borders, which also determines that the governance regime of cross-border data flow first started from the domestic data governance policies of countries and then gradually emerged at the level of international and regional organizations to regulate cross-border data flow through uniform data governance standards and model legal documents [8].

The article "Outbound Data Legality Analysis in CPTPP Countries under the Environment of Cross-Border Data Flow Governance" was retracted in 2023. Reasons: unreliable results or conclusions; concerns about the data; concerns about the results or conclusions; concerns about the peer review.

#### 2.1.2. Cross-Border Data Generation

Through the development of technology, humanity has once again crossed over from the “industrial age” to a new “digital age.” Digital information technology has transformed the volume of cross-border data flows from scarce to superabundant, and people live in a society where data and its impact are ubiquitous [9]. The value generated by cross-border data flows provided new impetus for global economic recovery and development.

*(1) Technology and the Times Give Rise to Cross-Border Data*. The generation of cross-border data has both a technical and contemporary background. From the technical side, the leap-forward changes in digital technology, the explosive growth of mobile terminals, inexpensive storage devices, high-speed broadband, and cloud computing are the prerequisites for cross-border data generation [10]. Digital technology involves all aspects of data generation, collection, and analysis. The automation of various digital image automatic collectors, chemical and biological sensors, data mining, data analysis, the increase of data storage capacity in the cloud, and the generation of data reading technology, graphic data conversion technology, and big data algorithms enable cross-border data to enter the stage of practical use. From the background of the times, cross-border data is generated in the current rapidly changing and developing digital environment. Every cross-border data generated currently will significantly impact the future, and these cross-border data are closely linked to the changing data environment. Quantitative decision-making based on data analysis will become increasingly popular [11]. The digital society has brought a new way of life to humanity, and the possibility and frequency of data interaction across borders have increased dramatically.

*(2) Diversified Uses to Expand Cross-Border Data*. In the “data age,” data has been integrated into all aspects of people's lives, and people's interactions constantly generate new data. In terms of usage, multinational enterprises first used cross-border data for market research, market analysis, and forecasting. Recently, the application of cross-border data has expanded to national foreign policy-making, regional economic cooperation, and regional human science research.

The article "Outbound Data Legality Analysis in CPTPP Countries under the Environment of Cross-Border Data Flow Governance" was retracted in 2023. Reasons: unreliable results or conclusions; concerns about the data; concerns about the results or conclusions; concerns about the peer review.

Cross-border data is access to a broader range of data at a lower cost. Cross-border data has a more comprehensive data universe, and predictive results based on such data are more valuable [12]. The predictive utility of cross-border data has emerged in economic development and public health.

With the expansion of cross-border data applications, cross-border data flow has become a cultural, commercial, and academic phenomenon. Culturally, cross-border online interaction among people in various countries has become a new socio-cultural and contemporary feature. Commercially, cross-border data provides a powerful source for international data analysis, prediction, and value mining for multinational enterprises. Academically, sociology, political science, and other humanities and social sciences have also started to use cross-border data to research particular topics.

The development of digital technology has promoted the full integration of data into people's lives, which in turn has caused cross-border data to be generated and begin to increase in large quantities. The increase of these data provides a vast space for mining its value, and this value space becomes the driving force for the uninterrupted flow and development of cross-border data later.

#### 2.1.3. Theory of Cross-Border Data Flow Governance

Along with the explosive growth of cross-border data, the digital economy is closely related to world trade and countries' core interests [13]. Although there is no unified governance regulation for cross-border data flow, most countries have adopted one of the following two governance theories for cross-border data governance: one is the “data sovereignty theory” based on the traditional sovereignty category; the other is the “data freedom theory” based on Internet cosmopolitanism. The second is the “data freedom theory” based on Internet cosmopolitanism [14].

*(1) Data Sovereignty Theory*. The encroachment of information technology on national sovereignty has been perceived since the sixteenth century. However, the emergence of printed publications at that time only affected and weakened governmental power. This information medium remained within the territory of the sovereign in physical space, where the supreme power could effectively control and dominate it [15]. However, with the development of modern information technology, the emergence of the Internet has significantly impacted the traditional theory of sovereignty [16]. The Internet's openness, boundarylessness, and virtual nature challenge the closed and exclusive concept of sovereignty. In this context, the concept of network sovereignty is created and has an essential impact on the theory of data sovereignty [17]. Therefore, the theory of data sovereignty mainly includes two connotations of network sovereignty and technological sovereignty.

The article "Outbound Data Legality Analysis in CPTPP Countries under the Environment of Cross-Border Data Flow Governance" was retracted in 2023. Reasons: unreliable results or conclusions; concerns about the data; concerns about the results or conclusions; concerns about the peer review.

On the one hand, since data is mainly transmitted through the network, the theory of data sovereignty is an extension of the theory of network sovereignty. In the existing theories, the definition of cyber sovereignty follows the lineage of traditional sovereignty and insists on the consistency of cyberspace and real space in international regulation. This is reflected in the “data sovereignty theory” of cross-border data governance, which holds that despite a series of new technological features of cross-border data flow, cross-border data governance should be subordinate to national sovereignty, and data sovereignty is the logical mapping of absolute sovereignty in the field of cross-border data governance. National governments have the right to independently and autonomously formulate cross-border data management regulations within their territories and rely on international institutions to realize the shared governance of cross-border data based on respecting the principle of sovereignty [18].

On the other hand, the development of technology is the root cause that allows cross-border data to be created, and the expansion of technological sovereignty has an essential impact on the theory of data sovereignty [19]. The EU first introduced technological sovereignty in the 2020 White Paper on Artificial Intelligence, a concept that emphasizes the need for the EU to own key data technologies and data infrastructures and reduce its dependence on others for data technologies; it also emphasizes that the EU should develop efficient mechanisms in data governance rules; and finally, it emphasizes that the primary purpose of technological sovereignty is to protect EU citizens and make “technology in the service of people.” Technological sovereignty mainly influences the data sovereignty theory of cross-border data governance from the technical, regulatory, and value levels [20].

*(2) Data Freedom Theory*. The second critical theory of cross-border data governance is the “data freedom theory,” based on Internet cosmopolitanism. Internet cosmopolitanism emphasizes the concept of a “world state” and believes that the Internet's virtual, open, and borderless nature makes cyberspace a space independent of reality, which can be freed from traditional sovereignty and form a “global commons” similar to the high seas and space. This space can be free from traditional sovereignty and form a “global commons” similar to the high seas and space, thus realizing a high degree of autonomy independent of the state. Influenced by this theory, the “data freedom theory” believes that the virtual, free-flowing, and nonexclusive technical characteristics of data can transcend the traditional concept of sovereignty and flow freely across borders without the control of state sovereignty, emphasizing that cross-border data governance should be managed in a weakly sovereign or even de-sovereign way [21].

The article "Outbound Data Legality Analysis in CPTPP Countries under the Environment of Cross-Border Data Flow Governance" was retracted in 2023. Reasons: unreliable results or conclusions; concerns about the data; concerns about the results or conclusions; concerns about the peer review.

The governance theory of “data freedom theory” is often placed in the context of economic or political unilateralism. The development of the digital economy is based on the free flow of data and the value of efficiency [22]. Suppose strong data localization regulations are made based on traditional sovereignty. In that case, it will inevitably hinder business development and act as a trade barrier, so sovereign intervention in cross-border data flow should be excluded as much as possible. The “data sovereignty theory” will hinder the cross-border flow of data and its value and efficiency and lead to the “balkanization” of the data field.

In summary, the “data sovereignty theory” is influenced by the concepts of network sovereignty and technological sovereignty and emphasizes the indispensable role of national sovereignty in data security and data development. In contrast, the “data freedom theory” emphasizes the free flow of data across borders as a driving force for the digital economy. The “data freedom theory” emphasizes the dynamics of the digital economy brought by the free flow of data across borders. The theoretical claims are closely related to the realistic demands. Various countries' cross-border data governance regulations are based on different interests in choosing different theoretical supports.

### 2.2. Legality of Data Exit Rules

The assessment of data export legality includes two aspects: legal and legitimate and risk-controlled. Lawful and legitimate include the following: First, it does not belong to the situation that laws and regulations explicitly prohibit the exit, such as the operation data of extensive national telecommunication facilities shall not leave the country; second, the exit of personal data shall obtain the authorized consent of the data subject; third, it is necessary to engage in normal business activities, fulfill contractual obligations, or fulfill legal obligations in China. For example, the cross-border e-commerce platform completes transactions by transmitting buyers' information. Travel agencies help customers book air tickets and overseas hotels during outbound travel; fourth, judicial assistance requires exit. Whether the data exit is risk-controlled is judged from the following two perspectives: first, the attributes of the data exit. Suppose the outbound data is large in volume, extensive in scope, sensitive, and not processed by security technology. In that case, it is likely to identify the sensitive information of individuals or a group by analyzing the potential connection between the data, which will seriously threaten the group's interests and national security, and second, the possibility of security incidents occurring in the outbound data. The following factors are included: (1) the technical and management capabilities of the sender's data exit. The sender needs robust data exit security monitoring technology, confidentiality processing technology, and data management technology to reduce the possibility of security incidents in cross-border data transmission; (2) the security protection capability of the data receiver. Only with this ability can the data recipient avoid leakage and loss of data upon arrival; and (3) the measures are taken and the political and legal environment of the country or region where the data recipient is located. After a security incident, both sides of the cross-border data transmission must take timely measures to avoid the continued expansion of adverse effects. At the same time, the political and legal environment of the data receiving party also has an important impact on the control of the consequences of harm and the relief of data rights.

The article "Outbound Data Legality Analysis in CPTPP Countries under the Environment of Cross-Border Data Flow Governance" was retracted in 2023. Reasons: unreliable results or conclusions; concerns about the data; concerns about the results or conclusions; concerns about the peer review.

### 2.3. Application of Machine Learning Algorithms in Legitimacy Assessment

#### 2.3.1. Overview of Machine Learning Algorithms

Machine learning incorporates knowledge from a variety of disciplines, a combination of disciplines that encompasses statistics, computer science, engineering, and more. As long as there is data interpretation in the field of data, there are machine learning algorithms [23]. Under the great wave of the Internet, the continuous development and innovation of big data and databases, more and more data can be saved, and different data begin to record all aspects of people's lives [24]. Facing such a vast amount of data, it would be significant to all aspects of human life if some algorithm or technology could be used to identify and understand the regular patterns in the data. Implementing machine learning is not just the simple use of computer algorithms, but these must be based on an accurate and complete data parsing [25].

#### 2.3.2. Implementation Process of Machine Learning Algorithms

*(1) Data Acquisition*. The critical steps of the process, which are broken down into data collection, preprocessing, model creation, and implementation, will still be followed by machine learning algorithms [26]. The application of issue solving will vary depending on the business settings [27].

*(2) Data Cleaning*. Data cleaning is the screening of data before analysis. In this study, cleaning the invalid, missing, and aberrant data typically consumes more than four-fifths of the time. Different algorithms also have slightly different data requirements [28].

*(3) Feature Engineering*. The feature vector tends to change with the needs of the model, and in general, researchers eliminate irrelevant or covariant features, and new features are generated as well [29]. Feature engineering significantly impacts the over- and underfitting of models and is a significant step in machine learning [30].

*(4) Model Construction and Optimization*. This procedure picks a model, tests it using the cleaned data, adjusts its parameters, and iteratively refines it until it has the best set of parameters based on the evaluation metrics it was chosen for [31].

*(5) Model Application*. The business department must verify and approve the optimal model before it can be used in practice. While it is being used in practice, the model's functioning and the data input and output must be examined for compliance [32].

The article "Outbound Data Legality Analysis in CPTPP Countries under the Environment of Cross-Border Data Flow Governance" was retracted in 2023. Reasons: unreliable results or conclusions; concerns about the data; concerns about the results or conclusions; concerns about the peer review.

## 3. Method

This paper uses a machine learning model to predict the legality of data exit from CPTPP countries. The text selected the outbound data from CPTPP countries as the study sample. A total of 100,000 outbound data were selected for the study as data and for training and validation, which cover different industries and fields and represent different countries of CPTPP.

### 3.1. Preparation Work before Model Building

#### 3.1.1. Construction of Derived Feature Variables

Derivative feature variables are new variables derived from the original feature variables through some calculations. The construction of derived feature variables is essential in the feature selection process. Derived feature variables can make the data exit legality evaluation index system more complete and reasonable. The construction of derived feature variables should be combined with the actual business situation and follow the corresponding principles.

In this paper, three derived feature variables are constructed for data exit legality based on the original feature variables based on experience and understanding of the business. After constructing the derived feature variables, 19 entry variables are finally determined.

#### 3.1.2. Standardization and Discretization Processing

*(1) Standardized Processing*. In model building, if the dimensionality of a feature is too large, it will significantly impact the similarity between samples, which will affect the model effect. Data standardization aims to solve the problem of dimensionality among the features. The features are comparable only after dimensionless processing, and the standard methods are Z-score standardization and Max-Min standardization [33].

The article "Outbound Data Legality Analysis in CPTPP Countries under the Environment of Cross-Border Data Flow Governance" was retracted in 2023. Reasons: unreliable results or conclusions; concerns about the data; concerns about the results or conclusions; concerns about the peer review.

Z-score normalization. Each sample is processed so the data has a fixed mean and standard deviation [34]. Specifically, it subtracted the overall mean *μ* from *f* and divided by the standard deviation *ρ*. It is expressed in the formula as *f*_*i*_′ = *f*_*i*_ − *μ*/*σ*.

Max-Min normalization. This is the process of mapping the sample *f* into [0, 1] for normalization, which is also a linear transformation of the original value interval of the sample to obtain a new interval [35]. The formula expresses it *f*_*i*_′ = (*f*_*i*_ − *f*_min_)/(*f*_max_ − *f*).

This paper uses the Z-score normalization treatment to normalize the continuous type feature variables (including derived feature variables). Z-score normalization transforms data of different magnitudes into the same magnitude uniformly and measures them uniformly with the calculated Z-score values to ensure comparability between data. In contrast, Z-score normalization transforms the data to have a mean of 0 and a variance of 1 without changing the distribution of the original data.

*(2) Discrete Processing*. When dealing with continuous data, it is necessary to discretize it for analysis. Data discretization processing means transferring finite samples in infinite space to finite space by means of mapping, improving the algorithm's spatio-temporal efficiency. In simple terms, discretization is the process of shrinking a dataset without changing its relative size. Effective discretization can decrease the algorithm's time-space overhead, enhance sample classification and clustering, increase the system's noise immunity, and successfully address data flaws that are hidden from view to increasing the model's stability. The standard data discretization methods are equidistant discretization and equal frequency discretization.

Equidistant discretization. According to the values of the continuous type attributes, they are uniformly divided into *k* intervals of approximately equal width, and the values of the attributes are correspondingly divided into the corresponding intervals to complete the discretization. The specific process is to use *f* to denote the continuous attributes to be discretized, calculate the width of the interval segment by the maximum and minimum values of the attributes: *w* = *f*_max_ − *f*_min_/*k*, and find the *k* − 1 cut points according to the obtained interval width w and the maximum value of the set of values, to complete the data discretization process.

The article "Outbound Data Legality Analysis in CPTPP Countries under the Environment of Cross-Border Data Flow Governance" was retracted in 2023. Reasons: unreliable results or conclusions; concerns about the data; concerns about the results or conclusions; concerns about the peer review.

Equal frequency discretization. In other words, the widths of the interval segments are no longer required to be consistent. The data volume of the discretized interval segments is balanced as much as possible by dividing them into *k* interval segments according to the total number of attribute values *n* so that the number of data contained in each interval segment is *n*/*k*. The value range of the data contained in each interval segment is the new discretized interval.

This paper uses the equal frequency discretization method because the qualitative features are initially discrete variables, so there is no need for discretization, and the continuous feature variables (including the derived feature variables) are discretized after normalization. The interval segment *k* is set to 5. Taking feature_one as an example, the distribution of this variable after discretization is shown in Figure 1.

#### 3.1.3. One-Hot Encoding Processing

For discrete feature variables such as “feature,” the numbers 1, 2, 3, and 4 are used in this paper to represent them, respectively. The value of these discrete features has no significance of size, but the introduced digital features bring order relations, which will affect the distance calculation between features. The introduction of one-hot coding can solve this problem. The introduction of one-hot encoding can solve this problem. In machine learning algorithms, calculating the distance between features or similarities is very important. Moreover, the commonly used calculation of distance or similarity is done in Euclidean space. By using one-hot encoding, we can extend the value of discrete features to the Euclidean space, and a value of discrete features corresponds to a point in the Euclidean space, which will make the distance calculation between features more reasonable. One-hot encoding, also known as one-bit valid coding, refers to the conversion of discrete fields with k values into *k* binary features with values of 0/1. It can be viewed as a representation of categorical variables as binary vectors. Introducing one-hot encoding also expands the features to some extent, as its values are only 0 and 1, and the different types are stored in the vertical space. The principle of one-hot encoding is shown in Figure 2.

Taking the feature variables as an example, the initial values of the variables are shown on the left, and the results of the variables after the one-hot encoding process are shown on the right, in the form of a two-dimensional matrix list. Since the continuous feature variables have already been discretized so that they also have the properties of discrete feature variables, the one-hot encoding process is applied to each feature variable under study in this paper.

The article "Outbound Data Legality Analysis in CPTPP Countries under the Environment of Cross-Border Data Flow Governance" was retracted in 2023. Reasons: unreliable results or conclusions; concerns about the data; concerns about the results or conclusions; concerns about the peer review.

#### 3.1.4. Partitioning the Training and Test Sets

The machine learning process is to train the created model with the data in the training set, then substitute the trained model into the test set to judge the model's performance, and finally decide whether the model can be used in real-life businesses. Therefore, dividing the training set and test set is an essential step in machine learning. In this paper, the illegal outbound data in the dataset is much less than the legal outbound data. To build a more objective outbound data legitimacy evaluation model, it should try to make the proportion of legal outbound data in the training and test sets consistent. This paper uses a stratified sampling method to divide the training and test sets. The process of dividing the training and test sets into three steps: stratification, random division, and merging, and the schematic diagram of the division method is shown in Figure 3.

This study divides the dataset into the training and test sets and sets the division ratio as 0.2. That is, 80% of the dataset is used as the training set, and 20% of the dataset is used as the test set. Moreover, the stratification is done according to the legality of the outbound data to ensure the repeatability of the division results. The results after the division are shown in Figure 4.

The results show that there are a total of 80,000 outbound data in the training set, of which 5,632 are illegal, and the illegal rate is around 0.07. There is a total of 20,000 outbound data in the test set, of which 1,387 are illegal. And the illegal rate is also around 0.07, which meets the requirement of stratified sampling and makes the construction of the legality prediction model of outbound data more objective later.

### 3.2. Modeling

The construction of the machine learning-based outbound data legitimacy assessment model is based on the theory of cross-border data governance, with the independent and dependent variables determined according to actual business needs. The core idea is based on the classification algorithm used by machine learning to solve the imbalance classification problem.

Machine learning classification algorithms include single classification algorithms and integrated classification algorithms. Single classification algorithms mainly include KNN, decision trees, and logistic regression; integrated classification algorithms include serial learner algorithm models and parallel learner algorithm models; and serial learner algorithm models include AdaBoost algorithm models, GBDT algorithm models, XGBoost, and parallel learner algorithm. The serial learner algorithm models include AdaBoost algorithm model, GBDT algorithm model, and XGBoost. The parallel learner algorithm models include the bagging algorithm and the random forest algorithm.

The article "Outbound Data Legality Analysis in CPTPP Countries under the Environment of Cross-Border Data Flow Governance" was retracted in 2023. Reasons: unreliable results or conclusions; concerns about the data; concerns about the results or conclusions; concerns about the peer review.

This papers use the logistic regression algorithm model and decision tree algorithm model in a single classification algorithm and random forest algorithm model and GBDT algorithm model in an integrated classification algorithm to construct the outbound data legitimacy assessment model.

#### 3.2.1. Modeling of a Single Classification Algorithm

*(1) Logistic Regression Modeling*. This study uses the logistic regression module in scikit-learn to build a logistic regression model. Firstly, the default logistic regression model parameters are used, and the divided training set is trained. The model is trained, then the test set is predicted, and the dichotomous labels are predicted, and it is found that the model is not practical. Therefore, it adjusted the parameters of the model, mainly the regularization parameter and the type weight parameter, and determined the optimal parameter penalty factor C to be 1.0, set the type weight parameter to be “balanced,” and assigned the weights according to the training sample size, and found that the model effect was significantly improved.

*(2) Decision Tree Modeling*. This study uses the decision tree module in scikit-learn to build a decision tree model. Firstly, the default model is used without adjusting the parameters, and it is found that the model is equally ineffective. Therefore, the parameters of the model are adjusted, mainly the maximum depth of the decision tree, the minimum impurity of node division, and the minimum number of leaf nodes samples. The method of adjusting the parameters is a combination of *K*-fold cross-validation and grid search method. The model is built and predicted, and the model effect is also found to be significantly improved.

#### 3.2.2. Modeling of Integrated Classification Algorithm

*(1) Establishment of Random Forest Model*. This study uses the random forest module in scikit-learn to build the random forest model. Firstly, the default parameters are used for prediction, and the model is less effective now. Then, the parameters are optimized. The main parameters are the number of decision trees, feature split evaluation criteria, the maximum depth of the decision tree, and the minimum number of samples required to split the internal nodes. Other parameters are set to default values.

*(2) GBDT Model Building*. This study uses the GBDT module in scikit-learn to build the GBDT model. Firstly, the default model is used for prediction, and it is found that the prediction effect of the model is poor. Therefore, the relevant parameters were set. The main parameters adjusted here were the number of decision trees, the maximum depth of decision trees, the minimum number of samples required to split the internal nodes, and the learning rate. In contrast, the other parameters were set to default values.

The article "Outbound Data Legality Analysis in CPTPP Countries under the Environment of Cross-Border Data Flow Governance" was retracted in 2023. Reasons: unreliable results or conclusions; concerns about the data; concerns about the results or conclusions; concerns about the peer review.

## 4. Results

### 4.1. Model Evaluation

The primary goal of the outbound data legitimacy assessment model is to distinguish legal outbound data from illegal outbound data, followed by the accuracy of the model prediction. Finally, the model also needs to have a certain degree of robustness. This paper uses AUC metrics to evaluate the accuracy of model prediction, KS metrics to evaluate the model's ability to identify whether the data are legal or not, and PSI metrics to evaluate the stability of the model's prediction for different samples. In addition, to prevent the model from overdetermining illegal outbound data as legal outbound data, recall, precision, and F1 scores are also introduced to ensure a more objective and comprehensive comparison of the models.

#### 4.1.1. AUC Indicators

In this paper, the logistic regression model is used as an example to calculate the AUC indicator, and the AUC value is the area under the ROC curve. The ROC curve and the AUC calculation results are shown in Figure 5. The AUC value of the logistic regression model is 0.84, which indicates that the logistic regression model has a high prediction accuracy in outbound data legitimacy assessment.

#### 4.1.2. KS Indicators

This paper takes the logistic regression model as an example to calculate the KS index. The KS indicator refers to Kolmogorov-Smirnov, which measures the difference between the cumulative good and lousy sample divisions. The more significant the cumulative difference between good and bad samples, the larger the KS indicator, and the better the model's ability to differentiate risk. The KS curve and the calculation results are shown in Figure 6. As can be seen from it, the KS value of the logistic regression model is about 0.5180, which corresponds to a threshold value of about 0.43. The KS value is more significant than 0.4, indicating that the logistic regression model can distinguish legal outbound data from illegal outbound data in the assessment of outbound data legitimacy.

#### 4.1.3. PSI Indicators

In this paper, the logistic regression model is taken as an example to calculate PSI index. Usually, PSI index is calculated using the data of different time periods, which is called “out-of-time test.” In this paper, because the data have no difference in time periods, the training set and test set are directly used to calculate, and the results are shown in Figure 7.

The article "Outbound Data Legality Analysis in CPTPP Countries under the Environment of Cross-Border Data Flow Governance" was retracted in 2023. Reasons: unreliable results or conclusions; concerns about the data; concerns about the results or conclusions; concerns about the peer review.

According to the results, it can be seen that the differences between the actual and expected percentages under each probability grouping are slight, reflecting a certain extent that the logistic regression model has good robustness in the assessment of the legitimacy of outbound data.

Finally, the PSI value is calculated using the custom function def in the following way.

(1) $$\begin{array}{c} \text{PSI}=\left({\left({\text{actual}}_{p}\text{rop}‐\text{expec}{\text{t}}_{p}\text{rop}\right)}^{*}\text{np}\cdot \log\left(\frac{{\text{actual}}_{p}\text{rop}}{{\text{expect}}_{p}\text{rop}}\right)\right)\cdot sum\left(\;\right), \end{array}$$

where *actual*_*prop* is the actual percentage and *expect*_*prop* is the expected percentage. The final calculated PSI value of the logistic regression model is 0.0051, and the PSI value is less than 0.1, which indicates that the logistic regression model has strong robustness in outbound data legitimacy assessment.

#### 4.1.4. Recall, Precision, and F1 Scores

This paper takes logistic regression model as an example to calculate recall, precision, and F1 score. The recall is specific to the original sample and indicates how many of the positive cases in the sample were predicted correctly. Precision is for our predicted results and indicates how many of the samples predicted to be cheerful are positive samples. The F1 score is the summed average of the precision and recall. The scores of recall, precision, and F1 under each threshold of logistic regression model were calculated. The higher the F1 score is, the better the comprehensive evaluation effect of the model is. In this paper, different thresholds are calculated, and the trends of precision, recall, and F1 score under different thresholds are plotted, as shown in Figure 8.

The precision of the logistic regression model increases with the increase of threshold, while the recall decreases with the increase of threshold, which again confirms the relationship between the two. That is, it is impossible to guarantee high accuracy in the case of a high recall rate. The F1 score first increased and then decreased with the threshold increase, reaching the maximum value of 0.3992 when the threshold was 0.8. For the legitimacy assessment of the outbound data in this paper, the threshold can be set as high as possible according to the actual demand; i.e., if the requirement for precision is high and if the requirement for the recall is higher, the threshold can be adjusted as low as possible. The F1 score is 0.3992, which corresponds to a threshold of 0.8; the recall is 0.3979, which is lower than the threshold of 0.5; and the precision is 0.4007, higher than the threshold of 0.5.

The article "Outbound Data Legality Analysis in CPTPP Countries under the Environment of Cross-Border Data Flow Governance" was retracted in 2023. Reasons: unreliable results or conclusions; concerns about the data; concerns about the results or conclusions; concerns about the peer review.

### 4.2. Model Comparison

The evaluation metrics of each logistic regression model, decision tree model, random forest model, and GBDT model were compared. The results are shown in Figure 9, where recall, precision, and F1 are the highest values calculated for each model at each threshold value.

All models showed sound effects with little difference in the scores of AUC, KS, PSI, and F1, among which AUC values were higher than 0.7, KS values were higher than 0.4, and PSI indexes were lower than 0.01. It shows that all the models have vital accuracy, robustness, and ability to distinguish the legality of outbound data.

The integrated classification algorithm model performs better in the AUC, KS, and F1 scores but has a smaller gap than the logistic regression model. In contrast, the decision tree model performs relatively poorly, and the decision tree performs best in the PSI index. For recall and precision, different models showed more significant differences, with the logistic regression model performing best on recall, the integrated model performing better on precision, and the decision tree model performing less well on both recall and precision.

### 4.3. Outbound Data Risk Score

The above models assess the legitimacy of outbound data, and the overall assessment effect is good. However, after all, it solves the problem of the dichotomous classification of outbound data legitimacy assessment without quantitative research on outbound data risk. This paper introduces an outbound data risk scoring model to quantify the risk of outbound data based on the determination of outbound data legitimacy and classifies the risk level of outbound data according to the score range for regulators to make a more scientific and reasonable judgment and thus make more complex decisions.

Since the purpose of outbound data risk scoring is to identify outbound illegal data as much as possible, and the logistic regression model performs best on recall, i.e., it is the best in identifying illegal outbound data, and this paper selects the logistic regression model as the base model to construct outbound data risk scoring.

#### 4.3.1. Outbound Data Risk Scoring

The outbound data risk score is a means to judge the likelihood of outbound data risk in the form of a specific score. The higher the score, the lower the likelihood of outbound data risk. The outbound data risk scoring model established in this paper uses the score's size to judge the data's outbound risk. The outbound data risk scoring model's final output is a score that is positively correlated with the probability of illegality.

The article "Outbound Data Legality Analysis in CPTPP Countries under the Environment of Cross-Border Data Flow Governance" was retracted in 2023. Reasons: unreliable results or conclusions; concerns about the data; concerns about the results or conclusions; concerns about the peer review.

The outbound data risk score is calculated as follows:

(2) $$\begin{array}{c} \text{score}=\text{BasePoint}-\beta \ln\left(\text{odds}\right), \end{array}$$

where the score is the final score, *BasePoint* is the benchmark score that has no practical significance, *β* is a constant that can be obtained by calculation, and odds are the ratio of the illegal probability of outbound data to the legal probability of outbound data, taking the logistic regression model of this paper as an example, assuming that the illegal probability of outbound data calculated by the logistic regression model is *p*, and then, the legal probability is 1 − *p*. That is, odds can be expressed as

(3) $$\begin{array}{c} \text{odds}=\frac{p}{1-p}. \end{array}$$

For the calculation of *β*, two assumptions need to be set as follows: (1) set a specific expected score for specific odds, i.e., set the expected score for odds of *θ* to *P*_0_ and the corresponding expected score for odds of 2*θ* to *P*_1_; (2) set the score for doubling odds (PDO), i.e., PDO = *P*_1_ − *P*_0_, indicating that the score increases by PDO units for each doubling of the good-bad ratio. Substituting into the formula (3), it can get

(4) $$\begin{array}{c} \begin{array}{c} P_{0}=\text{Base Point}-\beta \ln\left(\theta \right),\\ P_{1}=\text{Base Point}-\beta \ln\left(2\theta \right)\\ \text{PDO}=P_{1}-P_{0}. \end{array}, \end{array}$$

Solving for Equation (4) yields, the value of *β*

(5) $$\begin{array}{c} \beta =\frac{\text{PDO}}{\ln2}. \end{array}$$

In this paper, the value of PDO is set to 30. That is, for every doubling of the good to bad ratio, the score rises by 30 points, and *β* = 30/ln2 = 43.28 can be calculated, and base point is set to 500 points, and then, it can obtain the formula corresponding to the risk score of outbound data in this paper.

(6) $$\begin{array}{c} \text{score}=500-43.28\ln\left(\text{odds}\right). \end{array}$$

The odds can be obtained from the outbound data illegal probability *p* predicted by the logistic regression model.

#### 4.3.2. Outbound Data Risk Score Distribution

This paper uses a logistic regression model to predict the outbound data risk probability for the test set of outbound data and substitute the prediction results into (6) the formula to calculate the individual outbound data risk scores. After calculation, it is found that the highest outbound data risk score is 672, and the lowest outbound data risk score is 298 for the outbound data in the test set, with the score interval between [298, 672]. In general, the outbound data risk scoring model requires that the distribution of outbound data risk scores calculated for the same sample set is close to a normal distribution; otherwise, the sample set can be considered nonuniform, and the scoring results are not comparable. In this paper, histograms and kernel density plots are plotted for the outbound data risk scores calculated from the test set of outbound data to observe their distributions, as shown in Figure 10.

The article "Outbound Data Legality Analysis in CPTPP Countries under the Environment of Cross-Border Data Flow Governance" was retracted in 2023. Reasons: unreliable results or conclusions; concerns about the data; concerns about the results or conclusions; concerns about the peer review.

As seen from the result, the outbound data risk scores obtained by calculation of the test set are approximately normally distributed. The scores are mainly concentrated in the interval [450,600], indicating that this paper's outbound data risk score model is reasonable.

In this paper, the outbound data risk score obtained above is further divided into specific outbound data risk classes to provide more specific and clear decisions for outbound data regulators and a more detailed classification of outbound data risks. Specifically, the outbound data risk levels are classified according to the magnitude of the outbound data risk scores in different intervals, as shown in Figure 11.

As can be seen from Figure 11, the risk level of outbound data with a risk score greater than 600 is the high-risk level, which is the highest level. If outbound data is rated at this level, the probability of illegality of the outbound data will be very high, and it belongs to high-risk data. The risk level of outbound data with a risk score below 400 is no risk level, which is the lowest level, and the probability of illegality of such data is less than 1%. Data with risk scores between 400 and 600 are classified as low risk and medium risk, which should be released with caution and require a more in-depth assessment.

## 5. Discussion

There are still many areas for improvement in the process of risk assessment modeling of outbound data. In the preprocessing of data, this paper only adopts the oversampling method. It can also try the method of undersampling, the filling of missing values can try to fill with the plural or median or through algorithms, and it can also try other methods in the detection of outliers. Then, in the part of feature engineering, it can do some feature derivation. Secondly, it can also use the method of deep learning to create features to increase the model. The second is the deep learning method to create features to increase the model fit. Finally, in the model tuning, in this paper, only some parameters are selected for adjustment. To a certain extent, the accuracy of the model is affected. The article adopts different data mining tools, and through the comparison of multiple data models, the final generated outbound data risk assessment model has a more significant effect on the outbound data risk assessment, which can truly reflect the outbound data risk information and can effectively assist the establishment of the outbound data risk scoring system.

The article "Outbound Data Legality Analysis in CPTPP Countries under the Environment of Cross-Border Data Flow Governance" was retracted in 2023. Reasons: unreliable results or conclusions; concerns about the data; concerns about the results or conclusions; concerns about the peer review.

However, due to the limitations of research time, knowledge reserve, data collection, and information omission, this paper's outbound data assessment model is still imperfect. The first is that the data samples collected in this paper are not rich enough. Since the research of the article involves the acquisition of outbound data information, which is difficult to obtain, the quality of the available data is not high, and the data of essential indicators need to be fuzzy processed, all of which are true to different degrees, thus reducing the accuracy of the model. The second is that the assessment model in this paper relies on some subjective factors. This paper uses the data that the regulators have measured as the original data, which is inevitably influenced by the regulators' subjective factors. The information assessment of the outbound data will also form a specific deviation from the actual situation, thus causing the error of the model.

The model in the paper is only an initial establishment of the outbound data assessment model, which aims to analyze outbound data and assist in risk control. In the future, along with the improvement of the cross-border data flow system, the introduction of relevant laws, the establishment of an information resource sharing platform, and the enhancement of data security concept, data mining tools can play a more significant role in the prevention and control of outbound data risks.

## 6. Conclusion

This paper assesses the legitimacy of data exit rules of CPTPP countries based on machine learning algorithm models under the perspective of cross-border data flow governance. Four machine learning algorithms, logistic regression, decision tree, random forest, and GBDT, are used to build the outbound data assessment and evaluation models. Specifically, the confusion matrix is used to dichotomize the outbound data legality, and the parameters of each model are adjusted through regularization, cross-validation, and grid search. Then, the assessment metrics AUC, KS, PSI, recall, precision, and F1 scores are used to compare the empirical results of each model. Finally, based on this, it introduces a logistic regression-based outbound data risk scoring model to quantify the outbound data risk at a deeper level and classify the outbound data risk level for the reference of regulators to make more scientific and reasonable decisions. For outbound data legitimacy assessment, each machine learning model can meet the needs and applications of practical work and make accurate predictions. Its application in outbound data legitimacy assessment can provide a better reference basis for auditors; reduce human, material, and time costs; and has specific application prospects.

The article "Outbound Data Legality Analysis in CPTPP Countries under the Environment of Cross-Border Data Flow Governance" was retracted in 2023. Reasons: unreliable results or conclusions; concerns about the data; concerns about the results or conclusions; concerns about the peer review.

## Figures and Tables

**Figure 1:** Distribution of feature_one after discretization.

**Figure 2:** One-hot read thermal encoding principle.

**Figure 3:** Schematic diagram of stratified sampling.

**Figure 4:** Stratified sampling results.

**Figure 5:** ROC curve of logistic regression.

**Figure 6:** KS curve for logistic regression.

**Figure 7:** Logistic regression of actual vs. expected percentage.

**Figure 8:** Trend of precision, recall, and F1 scores.

**Figure 9:** Comparison of evaluation indicators by model.

**Figure 10:** Outbound data risk score distribution.

**Figure 11:** Outbound data risk level classification.

## Data Availability

The data used to support the findings of this study are available from the corresponding author upon request.
